# Online Troll Reviewer Detection Using Deep Learning Techniques

**DOI:** 10.1155/2022/4637594

**Published:** 2022-06-08

**Authors:** Mosleh Hmoud Al-Adhaileh, Theyazn H. H. Aldhyani, Ans D. Alghamdi

**Affiliations:** ^1^E-Learning and Distance Education, King Faisal University, Saudi Arabia, P.O. Box 4000 Al-Ahsa, Saudi Arabia; ^2^Applied College in Abqaiq, King Faisal University, P.O. Box 400, Al-Ahsa 31982, Saudi Arabia; ^3^Computer Engineering and Science Department College of Computer Science and Information Technology, Al Baha University, Saudi Arabia

## Abstract

The concentration of this paper is on detecting trolls among reviewers and users in online discussions and link distribution on social news aggregators such as Reddit. Trolls, a subset of suspicious reviewers, have been the focus of our attention. A troll reviewer is distinguished from an ordinary reviewer by the use of sentiment analysis and deep learning techniques to identify the sentiment of their troll posts. Machine learning and lexicon-based approaches can also be used for sentiment analysis. The novelty of the proposed system is that it applies a convolutional neural network integrated with a bidirectional long short-term memory (CNN–BiLSTM) model to detect troll reviewers in online discussions using a standard troll online reviewer dataset collected from the Reddit social media platform. Two experiments were carried out in our work: the first one was based on text data (sentiment analysis), and the second one was based on numerical data (10 attributes) extracted from the dataset. The CNN-BiLSTM model achieved 97% accuracy using text data and 100% accuracy using numerical data. While analyzing the results of our model, we observed that it provided better results than the compared methods.

## 1. Introduction

Antisocial behavior on social media can only be exposed if suspicious online reviewers are identified, as has been previously indicated. Antisocial behavior on the internet by trolls and other questionable reviewers can bring harm to web users and even potentially undermine democracy in some countries [1]. The problem is particularly serious because trolls actively spread hoaxes and misinformation during significant events such as elections or referendums. The purpose of this research is to develop a model that is effective in recognizing online trolls and to join forces with the multiple web platforms now trying to keep trolls at bay [2]. An important aspect of this study is the comparison of several approaches to machine learning and sentiment analysis in order to discover the most effective strategy in creating detection models for specific cases. For the sake of troll detection in diverse social networks, this research proposes to use deep learning approaches in model creation [3]. By examining the results of the comparison, we should be able to determine whether deep learning or sentiment analysis is preferable for building this detection model, as well as which approaches should be utilized for different types of text data and data from the structure of online debates.

In recent years, the advancement of information technology (IT) and internet-based apps has resulted in individuals all over the world generating vast amounts of data. Content is developed on a daily basis on a variety of online platforms, including social media status streams, films or photographs on e-commerce websites, and applications. People can share information and express their opinions and perspectives on products and services, as well as social issues, using social media, e-commerce websites, mobile platforms, and applications, among other media. Consumers' purchasing decisions are increasingly influenced by online product reviews [4], which are becoming more prevalent. Understanding the strengths and weaknesses of a company's goods and services through customer feedback is an effective approach in building enterprises, allowing business owners to capture what customers want and provide them with the best options. Exploiting and evaluating client product reviews has also become a competitive advantage for firms across a wide range of industries, particularly e-commerce websites.

Several different forms of trolls and dubious authors are associated with bogus accounts. Fake accounts have become quite popular in recent years, primarily because they allow for the manipulation of online web debates while remaining completely anonymous. As noted in one study [5], one or two posts are not enough to identify whether or not someone is a danger to a forum's community; rather, a person's complete profile must be scrutinized. Trolls frequently utilize postings in online discussions to disseminate phony reviews, spam, or connections to malicious websites that carry computer viruses. Different systems, such as troll-bots [6], can be used to generate spam and poisonous content on the internet. Automatic systems for recognizing and blocking suspicious reviews are being developed by web platforms. As a result, trolls frequently disguise harmful messages to make them more difficult to detect. For example, in a hostile atmosphere, they will not utilize foul or ugly language to hide their destructive content from automated systems. Additionally, masking can be achieved by purposefully generating mistakes in grammar or by exchanging letters in specific words. There is a need for comprehensive, emotional, and meticulously built lexicons [7] in order to meet this challenge.

Concerning suspicious includes any content that offends religious sensibilities; stokes antigovernment sentiments; incites terrorism; encourages illegal activities such as phishing, SMS, and pharming; or instigates a community without a legitimate reason [8–11]. As examples, social media was employed as a means of communication in the Boston Marathon bombing and during the Egyptian revolution [12]. The questionable content can be delivered in a variety of formats, including video, audio, pictures, graphics, and plain text. Text in particular is critical in this context, as it is the most extensively utilized mode of communication in cyberspace. Furthermore, by evaluating textual content, it is possible to determine the semantic meaning of a conversation, which is difficult to do with other types of content. Textual content analysis and classification into suspicious and nonsuspicious categories are the primary goals of this research.

A few previous studies have dealt with the issue of identifying toxicity in online comments written by individuals. Many of them use sentiment analysis techniques to identify and analyze subjective information to assess whether or not a toxicity feature is present [13–18]. Computational linguistics is the tools used most often for this purpose [19, 20]. Like many other machine learning techniques, sentiment analysis approaches may be divided into two primary types: supervised and uncontrolled. In order to develop a model that can be applied to unknown data, supervised approaches need to design the labeled data for training model [21, 22].

The vast amount of textual content on the internet makes it impossible to manually identify problematic texts [23]. As a result, it is necessary to create methods for automatically detecting questionable text content. Responsible authorities have been clamoring for a sophisticated tool or system that can detect questionable text messages. Such systems would also be useful in identifying potential cyber threats that are communicated through text-based content online. The automatic identification of suspicious text technology can quickly and accurately identify texts that appear questionable or menacing. Legislative and enforcement authorities can take necessary action promptly, which in turn serves to prevent virtual harassment as well as suspicious and criminal acts that are mediated over the internet. Due to the language's complicated morphological structure, vast number of synonyms, and numerous verb auxiliary variations based on subject, person, tense, aspect, and gender, categorizing Bengali text contents into suspicious or nonsuspicious categories can be difficult. Furthermore, the paucity of resources and the lack of benchmark datasets in Bengali make it more difficult to put into practice a suspicious text detection system than with other languages. According to the research questions asked in this paper [24], the main contributions of the developed system are as follows:

- Developing an integrated deep learning model for detecting troll reviewers in online discussion
- Testing the model using text data and numerical data
- Comparing the performance and results with existing methods
- Troll reviewers distribute misinformation to misguide readers into making wrong decisions in their daily activities; such misinformation includes fake news, rumors, and fake opinions

## 2. Background of Study

Instead of trolls or spam reviewers, a previous effort [25] focused on detecting an untrustworthy and fraudulent action known as phishing, employing a novel *K*-nearest neighbor (KNN) machine learning algorithm for detecting phishing assaults via URL classification. According to statistics from Kaggle, the best accuracy = 08.78% for phishing attack detection (*K* = 100). Overall, the proposed model has an accuracy of 0.858%. Spam reviewer detection was the focus of another paper [26], in which an unsupervised sentiment model based on Boltzmann machines was used to distinguish legitimate reviewers from spammers by supplying more text but using less relevant characteristics of an entity. This system was also trained to watch the progression of ideas over time, as spammers tend to focus for short periods of time to distort public opinion the most. Reputation fraud in product review data streams is the subject of the paper [27]. Dynamic programming was used by the authors to construct the most bizarre review sequences; conditional random fields were subsequently exploited to identify a review as legitimate or suspicious. The FraudGuard model was thoroughly tested as a result of these comprehensive studies.

Iskandar [28] collected data from social media sites such as Facebook and Twitter, and a variety of microblogging sites in order to train the model. They demonstrated that naive Bayes is the most appropriate algorithm for their work by doing a thorough examination of several algorithms [29–31]. It has been recommended that a technique for spotting suspicious social media accounts based on normalized compression distance be implemented. Jiang et al. [32] suggested future directions for determining suspicious behavior in various forms of communication. In a study utilizing machine learning techniques, the researchers and developers examined the originality of real and false news on 126,000 items that were tweeted 4.5 million times in total [33]. A proposed machine learning technique for recognizing hate speech in social media posts such as Twitter data has been presented in detail [34, 35]. Logistic regression with regularization exceeds other methods in terms of accuracy, achieving a 90% accuracy rating. In order to detect suspicious messages in Arabic tweets, an intelligent algorithm has been developed [35]. With a restricted set of data and classes, this system achieves a maximum accuracy of 86.72% by employing SVM techniques. With the use of a multiclass and binary classifier, Dinakar et al. [36] developed a method to analyze social media website like YouTube comments for the purpose of identifying textual cyberbullying. A unique technique for detecting Indonesian hate speech has been published which makes use of support vector machine (SVM), the lexical method, the word unigram method, and characteristics [37]. In this article [38], we will discuss a strategy for identifying abusive content and cyberbullying on Chinese social media. The authors obtained accuracy of 95% with their model, which was built with long short-term memory (LSTM) and considered the characteristics and behaviors of a client users [38]. Hammer [39] presented a method of identifying violence and threats from internet comments directed at minorities and other marginalized groups. The research looked at phrases that had been manually annotated and had bigram properties of key words.

For consumers on an e-commerce website, review language is one of the most straightforward and effective methods for expressing their feelings about a product, including their goals and motivation for making a purchase. As a result, it is important to investigate the sentiment expressed in these review texts. Many researchers have applied deep learning approaches that have demonstrated outstanding performance in other domains to emotive textual analysis [40]. The creation and optimization of neural networks [41] are the focus of the majority of current text classification research. According to Stojanovski et al. [42], who developed CNN-based method for sentiment analysis, the system has performs 8% better than standard sentiment analysis and sentiment identification of Twitter posts. A positional convolutional neural network (P-CNN) was suggested by Song et al. [43] that can enhance feature extraction by collecting positional properties at three distinct language levels: the word level, the phrase level, and the sentence level. Abdi et al. [44] developed a deep learning–based technique (RNSA) for sentiment analysis at the sentence level that employs recurrent neural networks (RNN) and LSTM to evaluate sentiment at the phrase level. Using multifeature fusion techniques, this methodology increased classification performance in review text sentiment classification by more than 5 percent when applied to review text sentiment classification. For document-level sentiment classification, Rao et al. [45] presented a novel neural network model (SR-LSTM) with two hidden layers to capture long-term context in texts and to make advantage of semantic linkages between phrases.

## 3. Materials and Methods

In this section, the framework for the used methodology for online troll reviewer detection is explained in details. It consists of various phases such as dataset collection, data preprocessing, splitting of the dataset, convolution neural network combined with long short-term memory technique (CNN-BiLSTM), and performance measurement metrics.  Figure 1 shows the workflow of the employed methodology in this study.

### 3.1. Dataset

For collecting datasets for this research, we used publicly available troll online reviewer dataset developed and created by Machova et al. [46]. This dataset have been collected from Reddit platform, and it concerned with online political discussion. As Reddit grows in popularity, many reviewers and users access this platform and there are number of suspected users. Reddit releases data on suspicious accounts and comments every year for scientific experiments. The distribution of the dataset is 10000 ordinary reviewer (nontroll reviewer) and 6695 troll reviewers. It consists of 12 attributes, which employed in two different experiments in this study.  Table 1 shows the description of the dataset attributes.

### 3.2. Data Preprocessing

The main objective of data preprocessing step is to make the data clean and free data noise. As we evaluated the dataset in two different experiments that using text data and other one is using numerical data for online troll reviewer detection. However, through preprocessing, the dataset was explored to find out if there are missing values within numerical attributes. According the exploration process, we found that the dataset have records with many missing values that have been dropped and the mean average is calculated instead of those values. For constructing CNN combined with the BiLSTM model for sentiment analysis score that was generated for troll reviewer detection, two attributes of the collected dataset which having text data were employed which are *Is_troll* and *Body.* Preprocessing steps such as stopwords removal, punctuations symbolic removal, emojis deleting, and tokenization (splitting given review text sentences into disconnected tokens or words) were applied on the body attribute, which the review text that is written by reviewer.

### 3.3. Data Splitting

In this phase, we divided the dataset into three sets: training, validation, and testing sets; then, the integrated convolutional neural network integrated with bidirectional long short-term memory (CNN-BiLSTM) model is applied to detect and classify the online troll reviewers in online discussion into troll or nontroll reviewer.  Table 2 below summarizes the results of data splitting process.

### 3.4. CNN-BiLSTM Model Description

Figure 2 illustrates the structure of the CNN-BiLSTM model for troll online reviewer detection. This model comprises of hidden neural network layers such as word embedding layer, convolutional layer, BiLSTM layer, and output layer.

#### 3.4.1. Word Embedding Layer

Before applying this layer, *N*-dimensional word representation vectors are created for each word of the reviews texts of the dataset using Word2Vect method. Mikolov et al. [47] have developed this method. An embedding layer employed in this model has constructed of three modules that are the vocabulary size (maximum features), embedding dimension, and input sequence length. We have specified each of these modules as vocabulary size into 20000 words, embedding dimension into 50 dimensions, and maximum length to 150 words. The process of mapping textual sentence of review text into numerical form is called as word embedding.

#### 3.4.2. Convolutional Neural Network

Deep learning techniques such as convolution neural networks (CNN) are used in a variety of fields, including text preprocessing, computer vision, and medical image processing [48, 49]. To retrieve the textual features from the input matrix created by embedding layer, the CNN-BiLSTM model uses a third layer called convolutional. In convolutional layer, 100 convolution filters are used to find the convolutions for each input sequence in input sentences matrix. Filter size was set into 3-dimensional matrix. The maximum pooling layer performs spatial dimensionality and downsampling. Input features in each filter kernel's pool are summed to get the maximum possible value.

#### 3.4.3. Bidirectional Long Short-Term Memory

Two hidden layers of dissimilar directions are connected to the same output in bidirectional LSTM networks. The BiLSTM network's production layer is able to acquire sequences of knowledge from both past and future states via the use of reproductive deep learning. Memory cells in the LSTM layer can ultimately distribute the outcomes of previous data features into the output layer. Furthermore, the learning of features occurs only in the forward direction, ignoring the backward connection and resulting in lower performance for the machine learning system. The bidirectional recurrent network technique processes data in both forward and backward directions to address this shortcoming. In every LSTM cell, four discrete computations are conducted based on four gates: input (*i*_*t*_), forget (*f*_*t*_),) candidate (*c*_*t*_), and output (*o*_*t*_). The equations for these gates are introduced and defined as follows:

(1) $$\begin{array}{c} f_{t}=\text{sig}\left({Wf}_{xt}+{Uf}_{ht}-1+b_{f}\right), \end{array}$$

(2) $$\begin{array}{c} i_{t}=\text{sig}\left({Wi}_{xt}+{Ui}_{ht}-1+b_{i}\right), \end{array}$$

(3) $$\begin{array}{c} O_{t}=\text{sig}\left({Wo}_{xt}+{Uo}_{ht}-1+b_{o}\right), \end{array}$$

(4) $$\begin{array}{c} c\sim t=\tanh\left({wc}_{xt}+{Uc}_{ht}-1+bc\right), \end{array}$$

(5) $$\begin{array}{c} C_{t}=\left(f_{\text{to}}ct-1+i_{\text{to}}c\sim t\right), \end{array}$$

(6) $$\begin{array}{c} h_{t}=O_{\text{to}}*\tanh\left(C_{t}\right), \end{array}$$

(7) $$\begin{array}{c} \tanh\left(x\right)=\frac{\;1-e^{2x}}{\;1-e^{2x}}, \end{array}$$

(8) $$\begin{array}{c} H_{t}=\left(\overset{⟶}{\;h_{t}}∶\overset{⟵}{\;h_{t}}\right), \end{array}$$

where sig and tanh are Sigmoid and tangent activation functions. *X* is the input data. *W* and *b* represent the weight and bias factor, respectively. *C*_*t*_ is cell state, *c* ~ *t* is candidate gate, *h*_*t*_ refers to the output of the LSTM cell, and $\left(\overset{⟶}{\;h_{t}}∶\overset{⟵}{\;h_{t}}\right)$ is concatenation output of forwarding and backward layer in LSTM.

#### 3.4.4. Classification Layer

A Sigmoid function is a final layer that performs detection and classification of the outputs classes (troll or nontroll reviewer). The sigmoid function equation is defined as follows:

(9) $$\begin{array}{c} \sigma =\frac{\;1}{\;1-e^{2x}}. \end{array}$$

### 3.5. Performance Measurement Metrics

In order to assess the proposed model CNN-BiLSTM, accuracy, precision, *F*1-score, and specificity metrics were employed. Equations of these performance measurements are presented below:

(10) $$\begin{array}{c} \text{Accuracy}=\frac{\text{TP}+\text{TN}}{\text{FP}+\text{FN}+\text{TP}+\text{TN}}\times 100\%, \end{array}$$

(11) $$\begin{array}{c} \text{Precision}=\frac{\text{TP}}{\text{TP}+\text{FP}}\times 100\%, \end{array}$$

(12) $$\begin{array}{c} F1‐\text{score}=2*\frac{\text{precision}\times \text{sensitivity}}{\text{precision}+\text{sensitivity}}\times 100\%, \end{array}$$

(13) $$\begin{array}{c} \text{Specificity}=\frac{\text{TN}}{\text{TN}+\text{FP}}\times 100\%, \end{array}$$

(14) $$\begin{array}{c} \text{Sensitivity}=\frac{\text{TP}}{\text{TP}+\text{FN}}\times 100\%, \end{array}$$

where True Pos (TP) indicate the total number of reviewers that are effectively identified and classified as nontroll reviewers. False Pos (FP) represents the total number of reviewers that are incorrectly classified as trolls. True Neg (TN) refer to the total number of reviewers that are correctly classified as trolls. False Neg (FN) denotes the total number of reviewers that are incorrectly classified as nontrolls.  Figure 3 shows the confusion matrices of the CNN-BiLSTM model for classification of online troll reviewers using text data (sentiment analysis) and numerical attributes, where the confusion metrics of CNN-LSTM approach is presented in Figure 4.

## 4. Experimental Results

This subsection presents the obtained results of two different experiments for classification of online troll reviewers using numerical data (10 attributes) and text data (sentiment analysis). The size of the dataset used in these experiments were 16695 samples divided as 70% as training, 10% as validation, and 20% as testing for the CNN-BiLSTM model. The first experiment was conducted for sentiment analysis of online reviewers was repeated 5 times in order to detect troll reviewers where the second experiment performed using numerical attributes and repeated 10 times in order to accomplish statistically significant results.  Table 3 shows the significant results of the experiments. The achieved results of these experiments were obtained on the respective testing sets.

As can be seen in above, the CNN-BiLSTM model achieved higher classification results using numerical data (10 attributes) than compared to text data.

### 4.1. Performance of Proposed System

A performance plot is known as learning curve that is a plot of model learning performance over the datasets. In these experiments, learning curves are used as diagnostic tool for measurement training and validation performance of the CNN-BiLSTM model that learned from the training dataset incrementally.  Figure 5 display the performance plots of CNN-BiLSTM models, where the performance of the CNN-LSTM models is shown in Figure 6.

As shown in above figures, the training performance of the CNN-BiLSTM model in case use of text data started from 84% and reach to 98%, and validation of the model was 97% where the model training and validation losses are reduced from 0.30 and 0.15 to 0.5 and 0.10, respectively.

## 5. Comparative Analysis

Table 4 summarizes the comparison results of the proposed model with existing methods using accuracy and the same dataset.

## 6. Conclusions

Deep learning model (CNN-BiLSTM) is proposed in this paper for detecting trolls in online discussions. Two separate experiments were carried out in this research work. Using numerical data for the first and text data for the second, as a result, when trained and tested on numerical data, the CNN-BiLSTM model performed better results than text data. Both experiments yielded satisfactory results using the model. These two types of data, text and numerical, are used in different ways to build detection model. Deep learning has an excellent job of processing text, but the training data that deep learning methods typically require is simply too large. As an experiment, it may be worthwhile to look into incorporating nontext data with text data into the model's training. From the experimental results, we observe that our model provide satisfactory results in all measurement metrics compared to the existing methods. In future, the advance deep leaning can be applied for improving the results.

## Figures and Tables

**Figure 1:** Workflow of the used methodology.

**Figure 2:** Structure of the CNN-BiLSTM model for troll reviewer detection using sentiment analysis.

**Figure 3:** Confusion matrix of CNN-BiLSTM using sentiment analysis.

**Figure 4:** Confusion matrix of CNN-BiLSTM using numerical attributes.

**Figure 5:** Performance plot of the CNN-BiLSTM model using text data.

**Figure 6:** Performance plot of the CNN-LSTM and model using numerical data.

**Table 1:** Description of the attributes of the used dataset.

Attribute name	Description
*Is-Troll*	Class labeling.
*Body*	This attribute indicates text based feature written and posted by the reviewer or user on Reddit portal.
*Score*	Sentiment polarity of the given comment text (-1 is negative and 1 is positive.
*Ups*	The number of like the reviewer has gotten on his/her comments and reviews texts through the Reddit platform.
*Down*	This attribute represents the number of dislikes received by the reviewer on his/her posts and comments.
*Link_karma*	This attribute is similar the comment karma. Conversely, link karma property does not expose the karma of the comments, but the karma of published posts of the user.
*Comment_karma*	In the Reddit forum, this property symbolizes the user's karma. Users who are rude, spamming, or spreading hoaxes are likely to have a lower karma than those who do not engage in such behavior.
*Has_verified_email*	If the user or reviewer has a verified email address, this characteristic is displayed. In the event that this address is not verified, it could imply that the author just set up the phony profile for the purpose of making troll posts and has since abandoned it.
*Is_gold*	There are two possible values for this attribute: 1 or nil. Users with accounts worth at least $1 are eligible for premium participation. Because premium membership on this network costs money, users who have it are less likely to be trolls.
*Controversiality*	Moderators on the Reddit platform are known for referring to hoaxes and controversial posts. The controversial characteristic means that the user has previously had a post rated as controversial. Moderators may have already flagged certain posts or comments from an account belonging to a persistent troll.

**Table 2:** Splitting of the used dataset.

Total number of samples	Training 80%	Validation 10%	Testing 20%
16695	12020	1336	3339

**Table 3:** Classification results of the CNN-BiLSTM model.

Type of experiment	Precision %	Sensitivity %	Specificity	*F*1-score%	Accuracy %
Experiment based on text data	0.99	0.922	0.993	0.955	0.97
Experiment based on numerical data	1.0	1.0	1.0	1.0	1.0

**Table 4:** Significant results of the CNN-BiLSTM against existing methods.

Models	Dataset	Accuracy %
SVM [1]	Numerical data	0.98
CNN [1]	Text data	0.95
Proposed CNN-BiLSTM	Numerical data Text data	1.0 0.97

## Data Availability

The dataset is available here: http://people.tuke.sk/kristina.machova/useful/
